RETRACTED

# The circRNA circAGFG1 acts as a sponge of miR-195-5p to promote triple-negative breast cancer progression through regulating CCNE1 expression

**DOI:** 10.1186/s12943-018-0933-7

**Published:** 2019-01-08

**Authors:** Rui Yang, Lei Xing, Xiaying Zheng, Yan Sun, Xiaosong Wang, Junxia Chen

**Affiliations:** 1 Department of Cell Biology and Genetics, Chongqing Medical University, #1 Yixueyuan Road, Chongqing, 400016 China; 2 Department of Endocrine and breast surgery, The First Affiliated Hospital of Chongqing Medical University, #1 Yixueyuan Road, Chongqing, 400016 China

**Keywords:** circAGFG1, miR-195-5p, Triple-nagetive breast cancer, CCNE1

## Abstract

**Background:**

In recent years, circular RNAs (circRNAs), a new star of non-coding RNA, have been emerged as vital regulators and gained much attention for involvement of initiation and progression of diverse kinds of human diseases, especially cancer. However, regulatory role, clinical significance and underlying mechanisms of circRNAs in triple-negative breast cancer (TNBC) still remain largely unknown.

**Methods:**

Here, the expression profile of circRNAs in 4 pairs of TNBC tissues and adjacent non-tumor tissues was analyzed by RNA-sequencing. Quantitative real-time PCR and in situ hybridization were used to determine the level and prognostic values of circAGFG1 in two TNBC cohorts. Then, functional experiments in vitro and in vivo were performed to investigate the effects of circAGFG1 on tumor growth and metastasis in TNBC. Mechanistically, fluorescent in situ hybridization, dual luciferase reporter assay, RNA pull-down and RNA immunoprecipitation experiments were performed to confirm the interaction between circAGFG1 and miR-195-5p in TNBC.

**Results:**

We found that circAGFG1 was evidently up-regulated in TNBC, and its level was correlated with clinical stage, pathological grade and poor prognosis of patients with TNBC. The results indicated that circAGFG1 could promote TNBC cell proliferation, mobility and invasion as well as tumorigenesis and metastasis in vivo. Mechanistic analysis showed that circAGFG1 may act as a ceRNA (competing endogenous RNA) of miR-195-5p to relieve the repressive effect of miR-195-5p on its target cyclin E1 (CCNE1).

**Conclusions:**

Our findings suggest that circAGFG1 promotes TNBC progression through circAGFG1/miR-195-5p/CCNE1 axis and it may serve as a new diagnostic marker or target for treatment of TNBC patients.

**Electronic supplementary material:**

The online version of this article (10.1186/s12943-018-0933-7) contains supplementary material, which is available to authorized users.

## Background

Breast cancer is one of the most popular malignant tumors among women and the second major cause of cancer-related deaths in women worldwide [1]. TNBC is the most malignant subtype of breast cancer accounting for approximately 15% of all breast cancers without expressions of estrogen receptor (ER), progesterone receptor (PR) and human epidermal growth factor receptor 2 (HER2). Compared with other breast cancer subtypes, TNBC occurs more frequently in young women, usually with a high histologic grade and poor prognosis [2]. Owing to defect of clear molecular markers, chemotherapy is the only available systematic therapy for TNBC. Although patients with TNBC could benefit from conventional chemotherapy, compared with other subtypes of breast cancer, this phenotype is associated with a higher distant recurrence rate and worse prognosis [3]. Therefore, it is urgent to discover novel molecular targets for therapy of TNBC patients.

RETRACTED

As a new type of endogenous non-coding RNA, circular RNAs (circRNAs) have the characteristics of a continuous covalently closed loop without the 5′-cap structure and the 3′-poly A tail [4]. Thousands of circRNAs have been discovered in mammalian cells with the development and integrated application of high-throughput sequencing technique and bioinformatics analysis. Although circRNA was considered as a by-product of a splicing error since it was firstly discovered in the cytoplasm of eukaryotic cells, nowadays it has been regarded as a pivotal regulator of a wide range of biological processes [5]. Recently, numerous of reports revealed that circRNAs are involved in the initiation and development of a variety of diseases, including cancers [6]. The circHIPK3, a well-known circRNA, was found to serve as a tumor suppressor in bladder cancer [7]. As another example, circFBLIM1 promoted hepatocellular cancer progression and may be a diagnostic biomarker and potential target for hepatocellular cancer therapy [8]. Some circRNAs were also identified as tumor suppressors or oncogenes in breast cancer [9, 10], however, circRNA associated with TNBC has rarely been reported up to date.

MicroRNAs (miRNAs) are small non-coding RNAs with a size of 18–25 nucleotides, which function as post-transcriptional regulators of target mRNAs [11, 12]. It is well known that the increase of oncogenic miRNAs expression in cancer leads to the downregulation of tumor-suppressive genes, whereas the decrease of tumor-suppressive miRNAs enhances the expression of oncogenes. The researches demonstrated that miRNAs can participate in tumorigenesis and progression of varies of cancers, including breast cancer [13–16]. However, the upstream regulators of miRNAs are poorly understood. Recently, Pandolfi et al. present a theory called the competing endogenous RNA (ceRNA) hypothesis that lncRNAs, mRNAs and pseudogenes could communicate with and regulate each other by competitively binding to the microRNA response elements (MREs), which provides a new mechanism of gene regulation [17]. It has been reported that circRNAs could also serve as ceRNAs to sequester away the miRNA from its target genes [18, 19]. CDR1as, acting as the most typical miRNA sponge, contains over 70 binding sites for miR-7 and intensely inhibited the miR-7 activity in neuronal tissues, resulting in increased levels of miR-7 targets [20]. However, biological functions of most circRNAs and the underlying mechanisms in pathogenesis and progression including TNBC remain largely unclear.

RETRACTED

Here, we first investigated the expression profile of circRNAs in TNBC using RNA-seq and identified a novel TNBC-related circRNA circAGFG1 from AGFG1 with a circBase ID of hsa_circ_0058514. Subsequently, we explored the clinical significance of circAGFG1 expression in TNBC, and gained insights into the function and underlying molecular mechanism of circAGFG1 in TNBC development and progression. The data showed that circAGFG1 was remarkably up-regulated in TNBC tissues and associated with clinical stage and pathological grade and positively correlated with CCNE1 expression. Up-regulation of circAGFG1 or down-regulation of miR-195-5p was closely related to poor prognosis of patients with TNBC. Further functional and mechanistic investigations revealed that circAGFG1 could promote cell proliferation and metastasis and inhibit cell apoptosis by acting as a sponge for the miR-195-5p to relieve microRNA repression for target gene CCNE1. Collectively, our data show that circAGFG1 might act as an oncogenic gene in TNBC progression and could be valuable marker and independent prognostic factor for TNBC diagnosis, therapy and survival.

## Methods

The 40 pairs of TNBC tissues and adjacent non-cancerous tissues including 4 pairs of samples for RNA-seq were collected from patients who were diagnosed with TNBC at the First Affiliated Hospital of Chongqing Medical University (Chongqing, China). All the patients have signed informed consent prior to surgery and did not suffer from other malignancy or receive preoperative chemotherapy or radiotherapy. Tissues were collected after surgical resection and stored in liquid nitrogen until further use. The present study was authorized by the Ethics Committee of Chongqing Medical University and conducted in conformity to the Declaration of Helsinki. The RNA-seq data of 116 TNBC and 11 adjacent non-tumor tissues and corresponding clinical data were obtained from The Cancer Genome Atlas (TCGA, https://cancergenome.nih.gov/).

RETRACTED

### Cell culture

Human TNBC cell lines (BT-549, MDA-MB-231, SUM-159, MDA-MB-453 and MDA-MB-468) and normal mammary epithelial cell line (MCF-10A) were purchased from American Type Culture Collection (ATCC) (Manassas, VA, USA). 293 T cell lines were preserved by our lab. MDA-MB-231, MDA-MB-453, MDA-MB-468, SUM-159 and 293 T cells were cultured in DMEM (Gibco, Carlsbad, CA, USA), BT-549 cells were cultured with RPMI 1640 (Gibco, Carlsbad, CA, USA), containing 10% fetal bovine serum, 100 U/mL penicillin and 100 mg/mL streptomycin. MCF-10A cells were cultured in MEBM BulletKit (Lonza, Basel, Switzerland). All these cell lines were maintained at 37 °C with 5% CO _2_ in a humidified incubator.

### RNA isolation, library synthesis and RNA sequencing

Total RNA was extracted with TRIzol reagent (Takara, Dalian, China) in accordance with the manufacturer’s protocols. The quality and quantity of isolated RNA were detected by Nanodrop 2000 spectrophotometer (Thermo Fisher Scientific, USA) and the integrity was examined by Agilent 2100 Bioanalyzer (Agilent Technologies, CA, USA). Purified RNA was treated with RiboZero rRNA Removal Kit (Epicentre, WI, USA) to deplete rRNA following the manufacturer’s protocols. The rRNA-depleted RNA samples were randomly fragmented into small pieces and synthesized cDNA with random primer. The PCR amplification products of cDNA were purified with AMPure XP Kit (Beckman Coulter, CA, USA). Then the libraries were quality controlled and sequencing of the libraries was performed with HiSeq2500 (Illumina, San Diego, USA).

### qRT-PCR

Total RNA was exacted and reverse transcribed into cDNA with PrimeScript RT Reagent Kit (Takara, Dalian, China) under recommended condition. qRT-PCR was conducted on a Bio-Rad CFX96 system (Bio-Rad, CA, USA) with TB Green Premix Ex Taq (Takara, Dalian, China). GAPDH was used as internal reference for quantification of circRNA and mRNA, while U6 for miRNA. The specific primers used are listed in Additional file 1**:** Table S1. The relative expression of genes was calculated by 2 ^–ΔΔCT^ method.

### Tissue microarray (TMA) and in situ hybridization (ISH)

The relative expression of circAGFG1 in TNBC tissues was detected by in situ hybridization with a specific digoxin-labeled circAGFG1 probe (Digoxin-5’-ATTTAATCCTCGCCTGCATGACTGTTGAAA-3′- Digoxin) (Geneseed, Guangzhou, China) on TMAs (Outdo Biotech, Shanghai, China) containing 80 paraffin-embedded TNBC samples. Concisely, after dewaxed in xylene and rehydrated through gradient alcohol, the TMAs were digested using proteinase K and hybridized with the specific circAGFG1 probe at 4 °C overnight, then incubated with anti-Digoxin-AP (Roche, Basel, Switzerland) at 4 °C overnight. The tissues were stained with NBT/BCIP (Roche, Basel, Switzerland) and quantified.

RETRACTED

### Vector construction and cell transfection

To overexpress circAGFG1, the full-length cDNA of circAGFG1 was amplified in 293 T cells and then cloned into over expression vector pLCDH-ciR (Geneseed, Guangzhou, China), which contained a front and back circular frame, while, the mock vector with no circAGFG1 sequence served as a control. To knock down circAGFG1, three siRNAs targeting the back-splice junction site of circAGFG1 and a siRNA-NC were synthesized by Geneseed (Guangzhou, China), after efficiency examination by qRT-PCR, siRNA-3 as the most effective one was used to construct siRNA plasmid vector (Additional file 2**:** Figure S1). Then the shRNA against circAGFG1 and negative control shRNA-NC were synthesized and cloned into pLL3.7 vector, named as sh-circ and sh-NC, respectively. All vectors were verified by sequencing. The miRNA mimics and inhibitors were purchased from GenePharma (Shanghai, China). Cell transfections were conducted with Lipofectamine 2000 (Invitrogen, Carlsbad, CA, USA) in accordance with the manufacturer’s protocols. The sequences of siRNAs and shRNAs were listed in Additional file 1**:** Table S2.

### Cell proliferation, cell cycle and apoptosis assays

The proliferation activity of TNBC cells was tested by Cell-Light™ EdU DNA Cell Proliferation Kit (Ribobio, Guangzhou, China) and Cell Counting Kit-8 (Bosterbio, Wuhan, China) following the manufacturer’s protocols, respectively. Colony formation assays were executed to determine the cloning capability of TNBC cells. Cell cycle analysis was implemented with PI staining by a flow cytometry (Becon Dickinson FACSCalibur, NY, USA). For apoptosis assays, TNBC and MCF-10A cells were harvested after transfection and double stained with fluorescein isothiocyanate (FITC)-conjugated Annexin V and propodium iodide (PI). Next, the percentage of early apoptotic cells was analyzed on a flow cytometer (Becon Dickinson FACSCalibur, NY, USA). Apoptosis was examined by One Step TUNEL (TdT-mediated dUTP Nick-End Labeling) Apoptosis Assay Kit (Beyotime, Shanghai, China) in accordance with the manufacturer’s protocols. TNBC and MCF-10A cells were fixed with 4% paraform for about 30 min, then stained with Hoechst 33342 (Beyotime, Shanghai, China) for 20 min and photographed under a fluorescence microscope (Leica, Wetzlar, Germany). Each experiment was repeated in triplicate.

### Wound healing and invasion assays

TNBC cells were seeded in 6-well plate and scratched with a 200 μL pipette tip in the middle of the wells at 24 h posttransfection, then cultured in serum-free medium. After 24 h, the width of wounds was examined in three-independent wound sites per group and normalized to control group. For invasion assays, 2×10^4^ TNBC cells were suspended in 200 μL serum-free medium after transfection and inoculated into the upper chambers (BD BioCoat, MA, USA) coated with matrigel (BD Biosciences, NJ, USA), and then 500 μL complete medium was added into the bottom chambers. After 24 h, the cells on the upper chambers were removed and cells on the lower compartment were fixed with ethanol and stained by crystal violet, then photographed and counted with a microscope (Leica, Wetzlar, Germany).

RETRACTED

### Animal experiments

All animal experiments were approved by Chongqing Medical University Animal Care and Use Committee and complied with the guidelines of the National Institutes of Health. Stably over-expressed cell lines were established by transfecting MDA-MB-231 cells with over expression and mock vector and selected with puromycin. MDA-MB-231 cells were infected with lentiviruses (Hanbio Co.LTD, Shanghai, China) carrying sh-NC and sh-circ, which termed LV-NC and LV-circ, respectively and selected with puromycin to obtain sh-circ or sh-NC stably expressed cell lines. For xenograft experiments, 2×10^6^ various kinds of MDA-MB-231 cells were subcutaneously inoculated into female BALB/c mice. The volume of tumors was measured once a week and calculated as 0.5×length×width^2^. The mice were sacrificed after 4 weeks and the tumors and lungs were removed for further analysis.

### Immunohistochemistry (IHC) and immunofluorescence (IF)

For IHC assay, paraffin sections were incubated with primary antibodies against CCNE1 (1:100), CDK2 (1:100), E2F1 (1:100) (Abcam, Burlingame, CA, USA) and pRB (1:100) (Cell Signaling Technology, Beverly, MA, USA) at 4 °C overnight, secondary antibodies at 37 °C for 1 h and HRP-labeled streptavidin solution for 10 min, then stained by diaminoaniline (DAB). For IF analysis, cell climbing pieces were incubated with antibodies against CCNE1 overnight at 4 °C and FITC-conjugated secondary antibodies, then dyed by DAPI and observed under a fluorescence microscope (Leica, Wetzlar, Germany).

### Fluorescence in situ hybridization (FISH)

FISH assay was executed to observe the location of circAGFG1 and miR-195-5p in TNBC cells. Briefly, after prehybridization at 55 °C for 2 h, frozen sections and cell climbing piece were hybridized with specific Cy3-labeled circAGFG1 probes (Cy3–5’-ATTTAATCCTCGCCTGCATGACTGTTGAAA-3’-Cy3) and FITC-labeled miR-195-5p probes (FITC-5’-GCCAATATTTCTGTGCTGCTA-3’-FITC) (Geneseed, Guangzhou, China) at 37 °C overnight, and dyed with DAPI. Slides were photographed with a fluorescence microscope (Leica, Wetzlar, Germany).

RETRACTED

### Dual-luciferase reporter assay

The sequences of circAGFG1 and CCNE1–3’UTR and their corresponding mutant versions without miR-195-5p binding sites were synthesized and subcloned into luciferase reporter vector psiCHECK2 (Promega, Madison, WI, USA), termed circAGFG1-WT, circAGFG1-Mut, CCNE1 3’UTR-WT and CCNE1 3’UTR-Mut, respectively. All these plasmids were validated by sequencing. The relative luciferase activity was examined by Dual Luciferase Assay Kit (Promega, Madison, WI, USA) in accordance with the manufacturer’s protocols.

### RNA immunoprecipitation (RIP)

RIP was conducted with Magna RIP kit (Millipore, Billerica, MA, USA) following manufacturer’s instruments. MDA-MB-231 cells were harvested 48 h after transfection of miR-195-5p mimics or miR-NC, and lysed in complete RNA lysis buffer, then cell lysates were incubated with magnetic beads which were conjugated with anti-Argonaute2 (AGO2) (Millipore, Billerica, MA, USA) or negative control IgG antibody (Millipore, Billerica, MA, USA) at 4 °C for 4 h. The beads were washed using washing buffer. Then immunoprecipitated RNA and protein were purified and enriched to detect the target RNAs and AGO2 by qRT-PCR and western blot.

### RNA pull-down

Biotin -labeled circAGFG1 probe (5’-GTGGTGGATTTAATCCTCGCCTGCATGACTGTTGAAATGT-3’-Biotin) and control probe (5’-CGACTTTGGCTTGTTCTGGCCTGCATGACTGTTGAAATGT- 3’-Biotin) were synthesized by Geneseed Biotech. MDA-MB-231 cells were lysed with lysis buffer and incubated with specific circAGFG1 probes. The cell lysates were incubated with streptavidin-coated magnetic beads to pull down the biotin-labeled RNA complex. The beads were washed and the complex was purified with TRIzol (Takara, Dalian, China). Then the abundance of circAGFG1 and miR-195-5p was analyzed by qRT-PCR.

### Western blot analysis

The total protein of TNBC cells was exacted with RIPA buffer and separated by 10% SDS-PAGE, then electransferred onto a PVDF membrane (Bio-Rad, CA, USA). The membranes were blocked with 5% skimmed milk powder and incubated with primary antibodies against CCNE1 (1:1000), CDK2 (1:1000), E2F1 (1:1000), CD44 (1:1000) (Abcam, Burlingame, CA, USA), RB (1:500), pRB (1:500), Bax (1:1000), Bcl-2 (1:1000), Caspase-3 cleaved (1:1000) and GAPDH (1:5000) (Cell Signaling Technology, Beverly, MA, USA) at 4 °C overnight and then incubated with secondary antibodies (1:5000) (Cell Signaling Technology, Beverly, MA, USA) at room temperature for 2 h. Finally, the bands were examined by Immobilob™ Western Chemiluminescent HRP Substrate (Millipore, Billerica, MA, USA).

### Statistical analysis

Statistical analyses were performed by SPSS 19.0 (IBM, SPSS, Chicago, IL, USA) and GraphPad Prism 5.0 (GraphPad Software Inc., CA, USA). Data were showed as mean ± standard deviation (SD). The differences between groups were assessed by Student’s *t* test, one-way ANOVA or χ^2^ test. The survival rates were evaluated by Kaplane-Meier method and tested by log-rank test. The effects of the clinical variables on overall survival of TNBC patients were determined by univariate and multivariate Cox proportional hazards regression model. The correlation between groups was analyzed by Pearson correlation. The diagnostic value was assessed with a receiver operating characteristic (ROC) curve. *P* value < 0.05 was considered as statistically significant.

RETRACTED

## Results

### circRNA and mRNA expression profiles in TNBC

In order to understand the expression profiles of circRNA and mRNA in TNBC, we applied RNA-seq in paired TNBC tissues and para-cancerous tissues from 4 patients with TNBC. With a cut-off criteria of fold change > 2.0 and *P* < 0.05, we found that a total of 354 circRNAs were differentially expressed between TNBC tissues and paired adjacent normal tissues, among which 47 were upregulated while 307 were downregulated (Fig. 1a). The 10 mostly increased and decreased circRNAs are depicted by heatmap (Fig. 1b). Notably, it was found that circAGFG1 (hsa_circ_0058514) was the most upregulated (15.04 folds) circRNA, which was spliced from AGFG1 located at chr2: 228356263–228,389,631 and finally formed a circular transcript of 527 nt according to the annotation of circBase (http://www.circbase.org/). Moreover, 3225 mRNAs were differentially expressed using the same cut-off criteria, including 1007 upregulated and 2218 downregulated mRNAs. And representative differentially expressed 20 mRNAs are displayed by heatmap (Fig. 1c). Kyoto Encyclopedia of Genes and Genomes (KEGG) enrichment analysis and Gene Set Enrichment Analysis (GSEA) were performed to investigate the function of mRNAs included in the expression profile. These two analysis results showed that cell cycle was the most significantly enriched pathway (Fig. 1d, e). CCNE1 was found to be the most upregulated (19.36 folds) cell cycle-related gene in TNBC tissues. As is known that cell cycle can act as a convergence point for oncogenic signaling pathways and aberrant cell cycle progression is a crucial characteristic of cancers. Hence, we focused our attention on circAGFG1 and CCNE1 in tumorigenesis and progression of TNBC in the present study.

**Fig. 1:** Expression profiles of circRNA and mRNA in TNBC. **a** The volcano plot visualizes the expression of circRNA between TNBC tissues and adjacent non-tumor tissues. The red dots and green dots represent upregulated and downregulated circRNAs with statistical significance, respectively. **b** and **c** The cluster heat maps displayed the 10 most increased and decreased circRNAs and representative differentially expressed mRNAs. Each column indicates a sample while each row indicates an individual circRNA or mRNA. The red and green strips represent high and low expression, respectively. **d** KEGG pathway analysis of differentially expressed mRNAs. **e** GSEA was performed in KEGG gene sets

RETRACTED

### circAGFG1 and CCNE1 are up-regulated in TNBC and associated with the progression and poor prognosis

To confirm the existence of circAGFG1, the cDNA of circAGFG1 was amplified in 293 T cells and verified by DNA sequencing. The results were in line with circBase (Fig. 2a). Then the expressions of circAGFG1 were detected in 40 pairs of TNBC tissues, TNBC cell lines (BT-549, MDA-MB-231, MDA-MB-453, MDA-MB-468 and SUM-159) and normal breast epithelial cells (MCF-10A) by qRT-PCR. In accordance with our RNA-seq data, the results showed that circAGFG1 were markedly upregulated in TNBC tissues and cell lines compared with adjacent non-tumor tissues and normal cell line (Fig. 2b, c). ROC analysis revealed that circAGFG1 could sensitively discriminate TNBCs from non-cancerous tissues (Fig. 2d). The relationship between circAGFG1 expression and clinical characteristics of the TNBC patients (cohort 1) were listed in Table 1. The expression of circAGFG1 is significantly correlated with T (*P* = 0.027) and N stage (*P* = 0.025). CircAGFG1 expression was then determined using ISH on TMAs which contained 80 TNBC tissues (Fig. 2e and f). The correlation between circAGFG1 expression and clinical characteristics of the TNBC patients (cohort2) were listed in Additional file 1: Table S3. Kaplan-Meier survival curve indicated that the expression levels of circAGFG1 were reversely correlated with overall survival of patients with TNBC (Fig. 2g). Further univariate and multivariate Cox regression analysis showed that TNM stage and circAGFG1 expression levels were independent prognostic factors for TNBC patients (Table 2).

**Fig. 2:** circAGFG1 and CCNE1 are up-regulated in TNBC and associated with the progression and poor prognosis. **a** PCR product of circAGFG1 in agarose gelelectrophoresis and the splicing site verified by DNA sequencing. **b** Relative expression of circAGFG1 in TNBC tissues (Tumor) and adjacent non-tumor tissues (Normal) was detected by qRT-PCR (*n* = 40). **c** Relative expression of circAGFG1 in cell lines was determined by qRT-PCR. **d** Diagnostic value of circAGFG1 for TNBC was evaluated by ROC curve. **e** Representative images of circAGFG1 expression in TNBC tissues were detected by ISH assays. Scale bar, 100 μm. **f** Percentages of specimen with low or high expression of circAGFG1 according to TNM stage. **g** Kaplan-Meier survival curve of overall survival in 80 patients with TNBC according to the circAGFG1 expression. Patients were stratified into high expression and low expression group by median expression. **h** Relative expression of CCNE1 in TNBC tissues (Tumor) and adjacent non-tumor tissues (Normal) was detected by qRT-PCR (*n* = 40). **i** Pearson correlation analysis of circAGFG1 and CCNE1 expression in 20 TNBC tissues. **j** Relative expression of CCNE1 in TNBC tissues (Tumor) compared with normal tissues (Normal) was analyzed using TCGA data. **k** Kaplan-Meier survival analysis of overall survival based on TCGA data (*n* = 103). Data were showed as mean ± SD, *P < 0.05, ***P < 0.001

**Table 1:** Correlation between circAGFG1 expression and clinicopathological features in 40 TNBC patients (cohort 1)

Characteristic		circAGFG1		Chi-square	*P* value
		Low	High		
		20	20		
Age	≥50	8	11	0.902	0.342
	< 50	12	9		
Menopausal	Premenopausal	11	7	1.616	0.204
	Postmenopausal	9	13		
Grade	II	14	10	1.667	0.197
	III	6	10		
T stage	T1	14	7	4.912	0.027^*^
	T2	6	13		
N stage	N0	12	5	5.013	0.025^*^
	N1-3	8	15		
TNM stage	I-II	18	15	1.558	0.212
	III	2	5		

^*^ *P* < 0.05

RETRACTED

**Table 2:** Univariate and multivariate Cox regression analysis of circAGFG1 and survival in patients with TNBC

Clinical variables	Univariate analysis		*P*	Multivariate analysis		*P*
	HR	95%CI		HR	95%CI	
Age (≥50 vs. < 50)	0.954	0.465–1.954	0.897			
Grade (II vs. III)	0.895	0.447–1.793	0.755			
T stage (T1 vs. T2/3)	1.048	0.505–2.176	0.889			
N stage (N0 vs. N1–3)	1.761	1.010–3.069	0.046^*^			
TNM stage (I-II vs. III)	2.296	1.141–4.620	0.020^*^	3.090	1.256–7.600	0.014^*^
circAGFG1 (low vs. high)	4.573	2.041–10.244	< 0.001^*^	6.072	2.614–14.105	< 0.001^*^

Abbreviations: *HR* hazard ratio, *CI* confidence interval

^*^P < 0.05

To ensure whether CCNE1 is co-overexpressed with circAGFG1, the levels of CCNE1 were examined in the 40 pairs of TNBC tissues and para-cancerous tissues by qRT-PCR. The results found that CCNE1 was also highly upregulated in TNBC (Fig. 2h). Pearson correlation analysis indicated that the expression levels of circAGFG1 were positively associated with those of the CCNE1 (Fig. 2i). Then, analysis of RNA-seq data of 116 TNBC tissues and 11 adjacent non-tumor tissues obtained from TCGA further confirmed that CCNE1 was upregulated in TNBC tissues compared with normal tissues (Fig. 2j). Further Kaplan-Meier survival curve analysis based on TCGA data showed that the higher level of CCNE1 was correlated with poorer prognosis (Fig. 2k). These results confirmed the robustness of our RNA-seq data and suggest that circAGFG1 and CCNE1 might participate in the tumorigenesis and development of TNBC.

RETRACTED

### circAGFG1 promotes TNBC cell proliferation

To explore the biological function of circAGFG1 in TNBC cells, the overexpression vector of circAGFG1 and the RNAi vector against circAGFG1 were constructed (Fig. 3a). The results showed that circAGFG1 was overexpressed and knocked down in MDA-MB-231 and BT-549 cells transfected with overexpression and RNAi vector using specific primers for circAGFG1 transcript by qRT-PCR (Fig. 3b). The qRT-PCR analysis demonstrated that both overexpression and knock-down experiments had no effect on the expression of linear transcript AGFG1 utilizing specific primers for linear AGFG1 (Fig. 3c). Growth curves performed by CCK8 assays demonstrated that upregulation of circAGFG1 significantly enhanced the proliferation viability of MDA-MB-231 and BT-549 cells, whereas downregulation of circAGFG1 inhibited cell growth (Fig. 3d). Similarly, EdU assays revealed that overexpression of circAGFG1 markedly increased the percentages of EdU-positive cells, while knockdown of circAGFG1 displayed an opposite effect (Fig. 3e, f). Colony formation assays further demonstrated that the cell cloning capabilities of MDA-MB-231 and BT-549 were significantly enhanced by upregulation of circAGFG1 and markedly impaired by downregulation of circAGFG1 (Fig. 3g, h). These experiments suggested that circAGFG1 enhances proliferation of TNBC cells.

**Fig. 3:** circAGFG1 promotes TNBC cell proliferation. **a** The schematic illustration of circAGFG1 expression vector and shRNAs. **b** and **c** qRT-PCR analysis of circAGFG1 and AGFG1 RNA expression in TNBC cells transfected with circAGFG1 expression vector, mock, sh-circ or sh-NC. **d** The growth curves of cells transfected with indicated vectors were evaluated by CCK8 assays. **e** and **f** EdU assays were conducted in cells after transfection with indicated plasmids (magnification, × 100). Scale bar, 100 μm. **g** and **h** Colony formation assays were executed to detect the proliferation of cells transfected with indicated vectors. Data were showed as mean ± SD, *P < 0.05, **P < 0.01, ***P < 0.001, N.S, nonsignificant

### circAGFG1 increases TNBC cell migration and invasion and modulates cell cycle and apoptosis

Then, wound healing and transwell assays were carried out to examine the effects of circAGFG1 on migration and invasion of TNBC cells. The results indicated that the migration and invasion abilities of MDA-MB-231 and BT-549 cells were markedly enhanced by upregulation of circAGFG1 but significantly suppressed by downregulation of circAGFG1 (Fig. 4a-d). We further evaluated whether circAGFG1 has an effect on cell cycle progression and apoptosis of TNBC cells. Cell cycle analysis revealed that knockdown of circAGFG1 led to higher percentages of MDA-MB-231 and BT-549 cells in G0-G1 phase as well as lower percentages of cells in S phase compared with control group, suggesting that downregulation of circAGFG1 resulted in G1 arrest of TNBC cells (Fig. 4e, f). Flow cytometry analysis with Annexin V/PI double staining showed that MDA-MB-231 and BT-549 cells transfected with sh-circ had a higher apoptotic rate than cells transfected with sh-NC (Fig. 4g, h). In addition, TUNEL assay showed that knockdown of circAGFG1 markedly elevated the number of TUNEL-positive cells compared with control group (Fig. 4i). Similarly, Hoechst33342 staining indicated that MDA-MB-231 and BT-549 cells transfected with sh-circ exhibited typical apoptotic morphology characteristics, including nuclear fragmentation, brighter fluorescent, chromatin condensation, apoptotic body and nuclear shrinkage (Fig. 4j). In addition, we further demonstrated that no changes in cell cycle and the number of apoptotic cells were observed in the circAGFG1 low-expression MCF-10A and SUM-159 cells lines transfected with the same sh-circ vector compared with control (Additional file 3: Figure S2). Furthermore, western blot was executed to detect the levels of apoptosis-related proteins. The results found that TNBC cells depleted of circAGFG1 had higher levels of proapoptotic protein Bax and activated (cleaved) caspase-3 as well as a lower expression of Bcl-2 compared with control group (Fig. 4k). These data suggested that circAGFG1 promoted the progression of TNBC cells in vitro.

RETRACTED

**Fig. 4:** circAGFG1 increases TNBC cell migration and invasion and modulates cell cycle and apoptosis. **a** and **b** Cell migration capacities were detected by wound healing assays after transfected with indicated vectors (magnification, × 50). Scale bar, 200 μm. **c** and **d** Cell invasion abilities were determined by transwell assays after transfection (magnification, × 100). Scale bar, 100 μm. **e** and **f** The cell cycle progression was analyzed by flow cytometry after transfected with indicated plasmids. **g** and **h** Apoptosis rate was analyzed by flow cytometry after downregulation of circAGFG1. **i** and **j** Apoptotic cells were assessed by TUNEL (magnification, × 100, scale bar, 100 μm) and Hoechst 33342 (magnification, × 200, scale bar, 50 μm) assays after knockdown of circAGFG1. **k** The expression levels of apoptosis-related proteins were determined by western blot. Data were showed as mean ± SD, *P < 0.05, **P < 0.01

RETRACTED

### circAGFG1 facilitates tumorigenesis, angiogenesis and metastasis of TNBC cells in vivo

To determine the effects of circAGFG1 on tumor growth and lung metastasis in vivo, MDA-MB-231 cells were stably transfected with over expression or mock vector and infected with LV-NC or LV-circ and then subcutaneously injected into female nude mice. As a result, the tumors derived from cells overexpressing circAGFG1 were bigger and heavier than those of the control group, and the tumors obtained from cells infected with LV-circ had smaller sizes and lower weights than tumors generated from cells infected with LV-NC (Fig. 5a-c). Moreover, upregulation of circAGFG1 could significantly promote tumors angiogenesis, while downregulation of circAGFG1 decreased the number of microvessels of the tumors compared with control tumors (Fig. 5d). In addition, overexpression of circAGFG1 led to a notable increase of metastasis nodes in the lungs of mice, whereas knockdown of circAGFG1 indicated a weak metastatic ability of the tumors compared with control group (Fig. 5e). Finally, to determine the effects of circAGFG1 on CCNE1 and downstream cell cycle related proteins, such as CDK2, pRB and E2F1, western blot and IHC staining of tumor tissues were executed in vivo. Western blot revealed that the expression of CCNE1 in circAGFG1 overexpressed tumor tissues was much higher than that in mock group, but the lower expression of CCNE1 was detected in circAGFG1 downregulated tumor tissues compared with the control group (Fig. 5f). IHC assay further demonstrated that upregulation of circAGFG1 could upregulate the expressions of CCNE1, CDK2, pRB and E2F1 in xenograft tumor tissues, in contrast, knockdown of circAGFG1 decreased the levels of these proteins (Fig. 5g). These results confirmed the oncogenic role of circAGFG1 in TNBC, suggesting that circAGFG1 might play a part in the regulation of cell cycle pathway.

**Fig. 5:** circAGFG1 facilitates tumorigenesis, angiogenesis and metastasis of TNBC cells in vivo*.* **a** Representative images of xenograft tumors of each group (*n* = 3). **b** Tumor weight was shown. **c** Growth curves of xenograft tumors which were measured once a week. **d** and **e** HE staining of tumor and lung sections displayed microvessels of the tumors and metastatic nodules of the lungs, respectively (magnification, × 100). Scale bar, 100 μm. **f** The protein level of CCNE1 was detected by western blot. **g** IHC staining was applied to analyze the protein levels of cell cycle-related molecules (magnification, × 200). Scale bar, 100 μm. Data were indicated as mean ± SD, *P < 0.05, **P < 0.01, ***P < 0.001

### circAGFG1 functions as a sponge for miR-195-5p

To elucidate the molecular mechanism underlying circAGFG1, firstly, we predicted the potential targets of circAGFG1 by miRNA target prediction software made by Arraystar according to TargetScan and miRanda database. The results showed that circAGFG1 possesses conserved target site of miR-195-5p with a high score (Fig. 6a). Considering that circRNAs could serve as miRNA sponges in the cytoplasm, we performed FISH assay in TNBC cells and tissues to observe the subcellular localization of circAGFG1 and miR-195-5p. It was found that most of circAGFG1 (red) and miR-195-5p (green) were co-located in cytoplasm (Fig. 6b, c). Then, the levels of miR-195-5p was examined in 40 pairs of TNBC tissues and adjacent non-cancerous tissues, the results indicated that miR-195-5p was markedly downregulated in TNBC tissues compared with adjacent non-tumor tissues (Fig. 6d). Furthermore, analysis of RNA-seq data from TCGA showed that miR-195-5p level in TNBC tissue (*n* = 115) was lower than that in normal tissues (*n* = 9) (Fig. 6e). Kaplan-Meier survival curve analysis based on the TCGA data exhibited a significant positive correlation between miR-195-5p expression and patients’ overall survival (Fig. 6f). Therefore, we supposed that circAGFG1 might serve as a ceRNA for miR-195-5p.

RETRACTED

**Fig. 6:** circAGFG1 functions as a sponge for miR-195-5p. **a** The miR-195-5p binding site on circAGFG1 predicted by targetScan and miRanda. **b** and **c** FISH was performed to observe the cellular location of circAGFG1 (red) and miR-195-5p (green) in cells (magnification, × 200, scale bar, 50 μm) and tissues (magnification, × 100, scale bar, 100 μm). **d** Relative expression of miR-195-5p in TNBC tissues (Tumor) and adjacent non-tumor tissues (Normal) was determined by qRT-PCR (*n* = 40). **e** Relative expression of miR-195-5p in TNBC tissues (Tumor) compared with normal tissue (normal) was analyzed using TCGA data. **f** Kaplan-Meier survival analysis of overall survival based on TCGA data (*n* = 100). **g** Schematic illustration of circAGFG1-WT and circAGFG1-Mut luciferase reporter vectors. **h** The relative luciferase activities were detected in 293 T cells after transfection with circAGFG1-WT or circAGFG1-Mut and miR-195-5p mimics or miR-NC, respectively. **i** and **j** Anti-AGO2 RIP was executed in MDA-MB-231 cells after transfection with miR-195-5p mimic or miR-NC, followed by western blot and qRT-PCR to detect AGO2 protein, circAGFG1 and miR-195-5p, respectively. **k** RNA pull-down was executed in MDA-MB-231 cells, followed by qRT-PCR to detect the enrichment of circAGFG1 and miR-195-5p. **l** The relative expression of miR-195-5p was detected by qRT-PCR after transfection with indicated vectors. **m** Pearson correlation analysis of circAGFG1 and miR-195-5p expression in 20 TNBC tissues. Data were indicated as mean ± SD, *P < 0.05, **P < 0.01, ***P < 0.001

In order to confirm the bioinformatics prediction analysis, dual-luciferase reporter assay was applied in 293 T cells. The full-length of circAGFG1-WT and mutant version without miR-195-5p binding sites were subcloned into luciferase reporter vector psiCHECK2 (Fig. 6g). The results indicated that miR-195-5p mimics could significantly decrease the luciferase activity of WT group but not mutant one (Fig. 6h), suggesting that there might be a direct interaction between circAGFG1 and miR-195-5p. It has been widely known that miRNAs regulate target gene expression by binding to Argonaute 2 (AGO2), the key component of RNA-induced silencing complex (RISC). Thus, an anti-AGO2 RNA immunoprecipitation (RIP) assay was conducted in MDA-MB-231 cells to pull down the RNA transcripts which bind to AGO2 with anti-AGO2 antibody, and IgG as a negative control. Indeed, AGO2, circAGFG1 and miR-195-5p were all efficiently pulled down by anti-AGO2 antibodies compared with IgG, moreover, both circAGFG1 and miR-195-5p were significantly enriched in cells transfected with miR-195-5p mimics compared with miR-NC group (Fig. 6i, j). To further verify the binding of circAGFG1 and miR-195-5p, we performed a circRNA pull-down assay with specific biotin-labeled circAGFG1 probes. Interestingly, a specific enrichment of circAGFG1 and miR-195-5p was detected by qRT-PCR in the circAGFG1 probe group compared with control probe (Fig. 6k).

RETRACTED

Additionally, we found that overexpression of circAGFG1 led to markedly decrease of miR-195-5p and silencing of circAGFG1 could significantly increase the expression of miR-195-5p in MDA-MB-231 and BT-549 cells (Fig. 6l). Pearson correlation analysis displayed a significantly negative correlation between the expression of circAGFG1 and miR-195-5p in 20 TNBC tissues (Fig. 6m). Collectively, these data demonstrated that circAGFG1 could act as a sponge for miR-195-5p in TNBC.

### CCNE1 is directly targeted by miR-195-5p and indirectly regulated by circAGFG1

According to the TargetScan (http://www.targetscan.org/vert_72/), CCNE1 and circAGFG1 share the same MRE of miR-195-5p. We conducted dual luciferase reporter assay to validate this prediction, the results showed that the activity of luciferase reporter vector carrying the CCNE1 3’UTR-WT sequence could be significantly decreased by miR-195-5p mimics compared with control groups (Fig. 7a, b). Moreover, miR-195-5p mimics could markedly reduce the expression of CCNE1, while miR-195-5p inhibitors significantly enhanced the level of CCNE1 in MDA-MB-231 and B-549 cells (Fig. 7c). As depicted in Fig. 7d, the protein levels of CCNE1 were accordingly altered in TNBC cells. To validate whether circAGFG1 could regulate the expression of CCNE1 in TNBC cells, we found that knockdown of circAGFG1 markedly decreased the expressions of CCNE1 and overexpression of circAGFG1 strongly increased the levels of CCNE1 (Fig. 7e). As expected, the increase or decrease of CCNE1 induced by circAGFG1 overexpression or knockdown could be reversed by miR-195-5p mimics or inhibitors, respectively (Fig. 7f). These data suggest that circAGFG1 could regulate the expression of CCNE1 through serving as a ceRNA for miR-195-5p in TNBC.

RETRACTED

**Fig. 7:** CCNE1 is directly targeted by miR-195-5p and indirectly regulated by circAGFG1. **a** Schematic illustration of CCNE1 3’UTR-WT and CCNE1 3’UTR-Mut luciferase reporter vectors. **b** The relative luciferase activities were detected in 293 T cells after transfected with CCNE1 3’UTR-WT or CCNE1 3’UTR-Mut and miR-195-5p mimics or miR-NC, respectively. **c** and **d** Relative mRNA and protein levels of CCNE1 were detected in cells after transfected with miR-NC, miR-195-5p, ihn-NC and inh-195-5p using qRT-PCR and western blot, respectively. **e** and **f** Relative expression of CCNE1 was detected by qRT-PCR in cells transfected with indicated vectors, miRNAs or inhibitors. Data were indicated as mean ± SD, *P < 0.05, **P < 0.01, ***P < 0.001

### circAGFG1 promotes TNBC cell proliferation and invasion through circAGFG1/miR-195-5p/CCNE1 axis

To explore whether circAGFG1 serves its biological function through circAGFG1/miR1–95-5p/CCNE1 axis, rescue experiments were designed using miR-195-5p mimics and inhibitors. The results indicated that the miR-195-5p mimics reversed the proliferation and invasion-promoting effects induced by overexpression of circAGFG1 in MDA-MB-231 cells, whereas miR-195-5p inhibitors could rescue the proliferation and invasion-suppressing effects of circAGFG1 knockdown in BT-549 cells by EdU and transwell assays (Fig. 8a, b). IF staining displayed that overexpression of circAGFG1 significantly increased the levels of CCNE1 and the effect could be abolished by miR-195-5p mimics, whereas downregulation of circAGFG1 reduced CCNE1 expression and the effect could be counteracted by miR-195-5p inhibitors (Fig. 8c). Furthermore, western blot demonstrated that upregulation of circAGFG1 enhanced the protein levels of CCNE1 and downstream targets CDK2, pRB, E2F1 and breast cancer stem cells marker CD44, while knockdown of circAGFG1 decreased the levels of these proteins and the effects caused by overexpressing or silencing circAGFG1 could be reversed by miR-195-5p mimics or inhibitors, respectively (Fig. 8d, e). In summary, these data demonstrated that circAGFG1 might serve as a ceRNA for miR-195-5p to regulate CCNE1 expression, which led to cell cycle out of control and development of TNBC (Fig. 8f).

RETRACTED

**Fig. 8:** circAGFG1 promotes cell proliferation and invasion through circAGFG1/miR-195-5p/CCNE1 axis. **a** and **b** The cell proliferation and invasion were determined after transfection with indicated vectors, miRNAs or inhibitors by EdU and transwell assays, respectively (magnification, × 100, scale bar, 100 μm). **c** Relative protein levels of CCNE1 in cells were assessed by IF after transfection (magnification, × 100, scale bar, 100 μm). **d** and **e** Relative expression of CCNE1 and downstream cell cycle-related molecules at protein level in cells transfected with indicated vectors, miRNAs or inhibitors was determined by western blot. **f** Schematic diagram of how circAGFG1 promotes TNBC tumorigenesis and progression. Data were indicated as mean ± SD, *P < 0.05, **P < 0.01, ***P < 0.001

## Discussion

In recent years, more and more circRNAs have been discovered in multiple tissues and cell lines by next-generation sequencing technology. Due to cell/tissue-specific and development stage-specific expression and molecular structure, circRNAs could possess regulatory function in various biological processes and they are better than linear transcripts as promising diagnostic markers or therapeutic targets for cancers [21]. Some circRNAs were reported to function as oncogenes or tumor suppressors in bladder cancer, gastric cancer, pancreatic cancer, hepatocellular carcinoma and other types of cancer [22–26]. To date, only a few circRNAs have been well functionally characterized and the biological function of most circRNAs remains largely unknown.

Here, we applied RNA-seq to obtain the expression profiles of circRNA as well as mRNA in 4 pairs of TNBC tissues and adjacent non-cancerous tissues. Subsequently, we identified a novel circRNA termed circAGFG1 which was obviously upregulated in TNBC tissues and significantly correlated with clinical stage and pathological grade as well as poor overall survival of patients with TNBC. Further, functional experiments in vivo and in vitro demonstrated that circAGFG1 significantly promoted proliferation and metastatic abilities of TNBC cells, while knockdown of circAGFG1 showed an opposite effect. Moreover, we explored the effect of circAGFG1 on stemness of TNBC cells in terms of CD44 expression level with western blot. The result showed that up-regulation of circAGFG1 could enhance stemness of TNBC cells by increasing CD44 expression, whereas circAGFG1 knockdown played a reverse role. It has been known that CD44 has been identified as a reliable marker for breast cancer stem cells and plays an important role in tumorigenesis, invasion and metastasis of TNBC [27]. These findings suggest that circAGFG1 acts as an oncogene in the progression of TNBC and it has the potential to become novel diagnostic and prognostic marker or therapy target for TNBC patients.

RETRACTED

The ceRNA hypothesis suggests that RNA transcripts, including mRNAs, lncRNAs, pseudogenes and circRNAs could crosstalk with and regulate expression each other via competing for shared miRNA response elements (MREs), building a new complicated post transcriptional regulatory network and mechanism [17]. Growing evidence indicated that some circRNAs could serve as sponges for miRNAs to regulate the expression of miRNA target genes in multiple human diseases including cancer. For example, it was reported that circRNA circCEP128 promoted bladder cancer development by functioning as a sponge for miR-145-5p to influence the expression of SOX11 [28]. Besides, circRNA circPRKCI promoted proliferation and occurrence of lung adenocarcinoma through sponging both miR-545 and miR-589 as a ceRNA and abated their suppression on the target gene E2F7 [29]. Moreover, circRNA hsa_circ_0052112 acts as sponge for miR-125a-5p to promote cell migration and invasion in breast cancer [30]. In our study, we found that circAGFG1 contained the MRE of miR-195-5p through bioinformatics analyses. FISH assay displayed that circAGFG1 and miR-195-5p were co-located in cytoplasm of TNBC cells and tissues. Therefore, we inferred that circAGFG1 might play an oncogenic role via sponging miR-195-5p in TNBC. Further, dual-luciferase reporter, anti-AGO2 RNA immunoprecipitation and RNA pull-down assays confirmed that circAGFG1 could interact with miR-195-5p directly. We still found that miR-195-5p was significantly downregulated in TNBC tissues and was positively correlated with patients’ overall survival with the TCGA dataset. Consistent with our results, it is reported that miR-195-5p is significantly downregulated in breast cancer patient tissues and cell lines and negatively correlated with the degree of malignancy of breast cancer [31]. Another study showed that miR-195-5p suppressed breast cancer proliferation, invasion and metastasis by targeting multiple genes [32]. MiR-195-5p is also found to be downregulated and may serve as a tumor suppressor for other cancers, such as prostate, lung and colon cancer [33–36]. Our findings demonstrated that circAGFG1 serves as an oncogene by sponging miR-195-5p in TNBC and revealed the significance of interaction between circAGFG1 and miR-195-5p in tumorigenesis and development of TNBC.

RETRACTED

According to ceRNA hypothesis, circRNA could act as a ceRNA to modulate the expression of miRNA target gene. We found that CCNE1, a vital cell cycle regulator, and circAGFG1 are co-overexpressed in TNBC. Interestingly, cell cycle was the most significantly enriched pathway according to GSEA and KEGG pathway analyses, which further support that cell cycle is closely related to tumorigenesis and development of TNBC [37]. Moreover, bioinformatics analysis indicated that CCNE1 is one of the potential targets of miR-195-5p using miRcode and TargetScan. Next, a dual-luciferase reporter assay confirmed that miR-195-5p could directly target the 3′-untranslated regions of CCNE1. Additionally, upregulation of miR-195-5p led to knockdown of CCNE1 at mRNA and protein levels, whereas downregulation of miR-195-5p displayed an opposite effect. It is known that CCNE1 mainly coordinates with CDK2 to regulate the cell cycle progression [38]. We found that down-regulation of circAGFG1 resulted in G1/S phase cell cycle arrest. The transcription factor E2F1 and the tumor suppressor protein retinoblastoma (pRb, RB) are 2 key regulators of cell cycle progression. Together they play roles in determining progression through checkpoints at G1/S and G2/M that dictate whether a cell can proceed with DNA replication and cell division. The CCNE1/CDK2 complex is able to phosphorylate RB and subsequently release and activate E2F1 transcriptional activity, pushing cell cycle from G1 to S phase, whereas dephosphorylation of RB promotes heterodimerization with E2F1 and suppression of E2F1 activity [39–41]. Our data suggest that circAGFG1 knockdown might inhibit the dissociation of E2F1 from RB due to changes of Rb phosphorylation mediated by CCNE1, which leads to decreased E2F1 transcriptional activity and G1/S phase cell cycle arrest. It is well-demonstrated that the dysregulation of CCNE1-CDK2 activity is implicated in multiple cancers, including bladder cancer, nasopharyngeal cancer and breast cancer [42–44]. It has also been demonstrated that overexpression of CCNE1 was related to poor prognosis in diverse of cancers [45]. Shaye and colleagues found that overexpression of CCNE1 is an early event in the progression of breast cancer [46]. The research revealed that overexpression of CCNE1 is a specific marker for TNBC [47]. Moreover, high level of CCNE1 was correlated with poor prognosis of breast cancer [48]. Consistent with former studies, we found that CCNE1 was significantly upregulated in TNBC tissues and overexpression of CCNE1 was correlated with shorter overall survival time. To validate the crosstalk between circAGFG1 and CCNE1, we uncovered that overexpression of circAGFG1 could increase CCNE1 in both mRNA and protein levels, while knockdown of circAGFG1 exhibited a reverse effect. Furthermore, these effects could be partially abolished by miR-195-5p mimics or inhibitors, respectively, which might support our hypothesis that circAGFG1 functions as a ceRNA to promote CCNE1-mediated proliferation and metastasis via decoying miR-195-5p in TNBC.

RETRACTED

## Conclusions

In conclusion, our results suggest that increased circAGFG1 expression is a frequent event and a potential independent prognosis marker for TNBC. We firstly demonstrated that circAGFG1 might sponge miR-195-5p to modulate CCNE1 expression, leading to tumorigenesis and development of TNBC. Our findings suggested that circAGFG1 could be a valuable prognosis marker and promising diagnosis and therapy targets for TNBC in the future. The regulatory network involving circAGFG1/miR-195-5p/CCNE1 axis might highlight a better understanding for potential mechanism of pathogenesis and progression of TNBC.

## Additional files

Additional file 1: **Table S1.** Sequences of primers used in this study. **Table S2.** Sequences of siRNAs and shRNAs used in this study. **Table S3.** Correlation between circAGFG1 expression and clinicopathological features in 80 TNBC patients (cohort 2). (DOCX 24 kb)

Additional file 2: **Figure S1.** The relative expression levels of circAGFG1 in 293 T cells transfected with indicated siRNA detected by qRT-PCR. *P < 0.05, **P < 0.01, ***P < 0.001, N.S, nonsignificant. (TIF 161 kb)

Additional file 3: **Figure S2.** The cell cycle analysis and apoptosis detection in the circAGFG1 low-expression MCF-10A and SUM-159 cell lines transfected with the same sh-circ vector. **(a)** The cell cycle progression was analyzed by flow cytometry. **(b)** Apoptosis was determined by flow cytometric analysis of Annexin-V/PI staining. **(c)** Apoptotic cells were assessed by TUNEL and Hoechst 33342 assays. N.S, nonsignificant. (TIF 680 kb)

## Abbreviations

3’UTR: 3′ -untranslated region
ceRNA: Competing endogenous RNA
CircRNA: Circular RNA
ER: Estrogen receptor
FISH: Fluorescence in situ hybridization
GSEA: Gene Set Enrichment Analysis
HER2: Human epidermal growth factor receptor 2
IF: Immunofluorescence
IHC: Immunohistochemistry
ISH: In situ hybridization
KEGG: Kyoto Encyclopedia of Genes and Genomes
miRNA: MicroRNA
PR: Progesterone receptor
qRT-PCR: Real-time quantitative polymerase chain reaction
RIP: RNA immunoprecipitation
RISC: RNA-induced silencing complex
RNAi: RNA interfere
RNA-seq: RNA sequencing
ROC curve: Receiver operating characteristic curve
TCGA: The Cancer Genome Atlas
TMA: Tissue microarray
TNBC: Triple-negative breast cancer
